# Expression of DNA Helicase Genes Was Correlated with Homologous Recombination Deficiency in Breast Cancer

**DOI:** 10.1155/2022/5508301

**Published:** 2022-07-09

**Authors:** Mengping Long, Hongjun Liu, Jinbo Wu, Shu Wang, Xin Liao, Yiqiang Liu, Taobo Hu

**Affiliations:** ^1^Department of Pathology, Peking University Cancer Hospital, Beijing, China; ^2^Department of Breast Surgery, Peking University People's Hospital, Beijing, China

## Abstract

Homologous recombination deficiency which is currently measured by the homologous recombination deficiency (HRD) score including score of telomeric allelic imbalance (TAI), large-scale transition (LST), and loss of heterozygosity (LOH) is highly related with sensitivity to platinum-containing drug and PARP inhibitors. DNA helicases are essential components for the homologous recombination repair process in which DNA helicases unwind double-strand DNA utilizing ATP hydrolysis. In our study, the correlation between the expression of DNA helicase genes and HRD score in breast cancer was analyzed. The overexpression in half of the DNA helicase genes was found to be highly correlated with a high HRD score both in BRCA-mutated and BRCA wild-type breast cancer. Moreover, HRD score can be predicted by a linear function contributed by five DNA helicase genes. In conclusion, our study revealed a close relation between the overexpression of certain DNA helicase genes and the deficiency of homologous recombination repair in breast cancer.

## 1. Introduction

DNA helicases are proteins that unwind DNA into single-strand structure utilizing the energy produced by ATP hydrolysis. They are also indispensable components in the repair process of DNA double-strand break (DSB) by homologous recombination repair (HRR) where the production of a single-strand DNA was essential [1]. Germline mutations in certain DNA helicase genes can cause cancer predisposition syndromes including the Bloom syndrome caused by *BLM* mutation [2] and the Werner syndrome caused by *WRN* mutation [3]. Moreover, the loss of function in DNA helicase genes including *RECQL*, *BLM*, *WRN*, *RECQL5*, and *BRIP1* are also known to be highly correlated with the carcinogenesis of breast cancer and the BRCAness phenotype in breast cancer [4–8].

In breast cancer, the deficiency in homologous recombination repair pathway is called “BRCAness phenotype” and can be measured by the presence of genomic scar including telomeric allelic imbalance (TAI), large-scale transition (LST), and loss of heterozygosity (LOH) via single nucleotide polymorphism (SNP) profile. The numeric sum of the TAI, LST, and LOH is called HRD score, and a HRD score greater than or equal to 42 is defined as BRCAness phenotype. BRCAness phenotype in breast cancer has been shown to be highly correlated with the response to platinum-based chemotherapy and PARP inhibitors in *BRCA1* and *BRCA2* germline wild-type triple negative breast cancer (TNBC) [9, 10]. Importantly, in BRCA wild-type TNBC, the percentage of BRCAness phenotype was shown to be over 50% [9] even though the mechanism for the specific cause of HRD was unclear in those samples. Thus, it is important to characterize the molecular features of breast cancer with BRCAness phenotype in order to understand the detailed mechanism and to develop a more convenient biomarker for the evaluation of HRD.

Previous studies have focused on the mutation of targeted genes in the HRR pathway, while numerous recent papers have shown that the altered expression in DNA helicase genes including *BLM*, *RECQL5*, *SLFN11*, and *ATM* have impact on the HRR efficiency and consequently sensitivity on platinum-based chemotherapy and PARP inhibitors [11–14]. Also, studies showed that small molecules inhibiting DNA helicases including BLM and WRN could induce DNA damage and sensitivity to PARP inhibitor [15, 16]. Thus, it provides the rationale for us to look at the effect of the expression of DNA helicases which are essential components in the HRR pathway on the measured HRD status in breast cancer. In this study, we comprehensively analyzed the correlation between the expression of DNA helicase genes participated in HR and the HR status in breast cancer defined by the HRD score using TCGA data. A strong correlation between the overexpression of DNA helicase genes and HRD was find both in *BRCA1/2*-mutated breast cancer as well as in *BRCA1/2* wild-type breast cancers. A gene signature composed of five DNA helicase genes was identified that can predict the HRD score with high accuracy.

## 2. Materials and Methods

### 2.1. Data Collection

Data acquisition and analysis were conducted using R software (version 3.5.1 or above) unless otherwise mentioned. RNA-seq and clinical data were downloaded from the TCGA dataset [17] using the TCGAbiolinks R/Bioconductor package (version 2.10.5) [18]. The three genetic signature scores and HRD score of breast cancers from TCGA were derived from previous study, together with the germline mutation status of BRCA1/2 genes [10]. The genetic signature score is calculated using algorithms developed by researchers using the Affymetrix SNP6 data downloaded from TCGA.

Fragments per kilobase of transcript per million mapped reads upper quartile (FPKM-UQ) is used for the normalization of RNA transcript reads. FPKM-UQ RNA-seq data were downloaded and prepared using the GDCquery, GDCdownload, and GDCprepare functions, as described in our previous publications [19–21].

### 2.2. Correlation Heatmap Generation

Unsupervised hierarchical clustering and heatmap generation was performed using “ComplexHeatmap” package. Comparison of HRD scores and gene expression values between different groups was performed by Students' *t*-test. *P* values were calculated as two-sided, with statistical significance declared for *P* less than 0.05.

### 2.3. Correlation Analysis and Model Building

The best multivariate model was generated using the “bess” function from “BeSS” R package. The “BeSS” package uses primal dual active set (PDAS) algorithm to solve the best subset selection problem under the general convex loss setting. The algorithms can be used for variable selection in a linear model. The correlation analysis between predicted HRD and actual HRD score was evaluated with Pearson's correlation coefficient.

## 3. Results

### 3.1. The Expression of DNA Helicase Genes Was Positively Correlated with HRD Score in Breast Cancer

871 cases of breast cancer patients were included in the study, and the scores of genomic scars including TAI, LST, and HRD-LOH were obtained from previous study [10]. *BRCA1* or *BRCA2* germline mutation was found in 43 of them with 23 patients harboring pathogenic mutations and the others harboring nonpathogenic mutations [10]. The threshold for defining HRD score high and low was based on the average HRD score in BRCA pathogenic mutation population which was 58.9. Thus, a HRD score ≥ 59 was considered HRD high and a score smaller than 59 was considered to be HRD low. This HRD threshold score is set higher than the conventional threshold of 42. Twenty-two DNA helicase genes participating in homologous recombination were analyzed in the study. The correlation between the expression of DNA helicase genes and HRD score was calculated and a correlation heatmap was generated (Figure 1). The scores of TAI, LST, and LOH were highly correlated with each other as they show very similar correlation with each gene. The 22 DNA helicase genes were clustered by K-means algorithm and can be divided into 4 groups according to their correlation with HRD score (Figure 1). Among them, the expression of *BLM*, *PIF1*, *POLQ*, and *PARPBP* showed highly positive correlation with HRD score which was included in group 4. Six out of the 22 genes were included in group 3 which showed modest positive correlation with HRD score, and three of them in group 1 showed modest negative correlation with HRD score. No significant correlation was observed between the other nine genes and HRD score. Among the 22 selected DNA helicase genes, the expression of *SLFN11* has been previously shown to be correlated with homologous recombination efficiency and drug sensitivity to PARP inhibitor in non-small-cell lung cancer [11–13], while no correlation was detected between *SLFN11* expression and HRD score in breast cancer by this study.

### 3.2. Overexpression of DNA Helicase Genes Contributed to Both BRCA-Related and -Unrelated HRD

Next, the correlation between gene expression and HRD score was analyzed in BRCA-mutated and nonmutated patients. Breast cancer with pathogenic germline BRCA mutation harbored high HRD score when compared with BRCA wild-type and nonpathogenic mutation group (Figure 2). No difference was identified between nonpathogenic mutation group and wild-type group. However, for BRCA wild-type breast cancer, there were also 17.5% (145/828) of them having a HRD score above the average of BRCA mutated breast cancer, while no specific genetic mutation can be attributed to explain the mechanism. When the correlated DNA helicase genes identified above were analyzed, it was found that all of the positively correlated genes except *RECQL4* showed higher expression in HRD high patients regardless of BRCA mutation status (Figure 3), whereas for the three negatively correlated genes, lower expression was noticed in HRD high group only in BRCA wild-type cases. No difference in expression was identified between BRCA-mutated group and HRD low group. The above results indicated a shared mechanism behind HRD-high groups caused regardless of BRCA mutation status.

### 3.3. Gene Signature of DNA Helicase Genes Can Predict the Status of HRD in Breast Cancer

We next further explored the possibility of predicting HRD score using the expression of DNA helicase genes. A linear regression model was built to predict the HRD score of each breast cancer using the above DNA helicase genes. The model was represented as following:

(1) $$\begin{array}{c} \text{HRD}=4.52\times \text{BLM}+5.40\times \text{FIGNL}1+4.72\times \text{PIF}1+10.31\times \text{FBXO}18–8.78\times \text{HELQ}-227.56. \end{array}$$

Using this model, the predicted HRD score has a correlation score of 0.64 with the actual HRD score (Figure 4). Thus, our study built a new model for the prediction of PARP inhibitor efficiency in breast cancer as shown in Figure 5. In breast cancer patients with germline pathogenic BRCA1/2 mutations, cancer cells harbor homologous recombination repair deficiency (HRD) due to malfunction of BRCA1 or BRCA2 protein in DNA damage repair. The application of PARP inhibitors in these patients causes defect in single-strand DNA damage repair due to inhibition of PARP-1 protein. The block of both repair pathways promotes the apoptosis of tumor cells, which is called the “synthetic lethal” mechanism of PARP inhibitors, while for breast cancer patient without pathogenic BRCA1/2 mutations, HRD score can be predicted with gene expression of five DNA helicase genes using the linear regression model to further select breast cancer patients with HRD phenotype. When the predicted score is greater than 0.64, the possibility of HRD should be considered and this part of breast cancer could possibly benefit from the treatment of PARP inhibitors.

## 4. Discussion

In this study, the correlation between the expression of DNA helicase genes and the HRD score was analyzed. A strong correlation between the overexpression of DNA helicase genes and HRD was found both in *BRCA1/2*-mutated breast cancer as well as in *BRCA1/2* wild-type breast cancers. And a linear model was built to predict the HRD score using the mRNA expression of five DNA helicase genes with high accuracy. The correlation between the overexpression of DNA helicase genes and HRD in breast cancer has been reported before. Previous studies found that overexpression of BLM can promote the occurrence of DNA damage and the knockdown or deficiency of BRCA1 induced the overexpression of *BLM*, indicating the role of *BLM* in both BRCA1-related and -unrelated homologous recombination repair [22]. However, our study reported for the first time that the overexpression in multiple DNA helicase genes was highly correlated with HRD indicating a shared mechanism among them. Further studies need to be conducted to reveal the exact molecular mechanism.

PARP inhibitors including olaparib, rucaparib, niraparib, and talazoparib have shown robust efficiency in breast cancer patients with germline BRCA1/2 mutation both as second-line therapy and as first-line therapy [23–25]. Moreover, molecular and early clinical study demonstrated that PARP inhibitor was also effective in BRCA1/2 wild-type cells with HRD phenotype [26, 27]. However, the measurement of HRD score was currently expensive and inconvenient compared with measurement of gene expression. Our study showed that HRD score in breast cancer can be effectively predicted by the expression of DNA helicase genes which provided a tool for assessing BRCAness phenotype in breast cancer. Despite PARP inhibitors, other small molecules targeting the HRR pathway through DNA helicase proteins in breast cancer have been developed as potential therapeutics. A small molecule which binds specifically to DNA helicase RECQL5 and stabilizes the interaction between RECQL5 and RAD51 could inhibit the proliferation of breast cancer cells in a RECQL5-dependent manner [28]. Noticeably, the above study is performed in MCF-7 cell line which has wild-type BRCA1/2 gene, suggesting that the HRR pathway could also be a target in BRCA1/2 wild-type breast cancer. Also, study showed that using CHK1 inhibitor in WRN-deficient cancer cells could produce synergic killing effect [29, 30]. Together with the results in our study, the expression of DNA helicase could be a tool of measuring HRR status as well as a therapeutic target in breast cancer.

Our study is limited by the fact that the developed model has only been tested in a single database. Validation in other breast cancer database should be performed in future work. Besides, this model may be experimentally validated to show HR deficiency in cancer, as mentioned by various methods in many recent reports, for instance, a recent study evaluated response of PARP inhibitor using autophagy-proficient and -defective breast cancer cells and xenograft SCID-mice model [31]. Future validation of our work could be performed by constructing breast cancer cell lines overexpressing DNA helicases *BLM*, *FIGNL1*, *PIF1*, or *FBXOI8* and cell lines downregulating *HELQ*. Efficiency of HRR in the constructed cell lines should be evaluated by assays including H2Agamma foci quantification. Sensitivity to PAPR inhibitor should be evaluated.

## Figures and Tables

**Figure 1:** Correlation heatmap between the expression of DNA helicase gene and the score of genomic scars. The correlation efficiency between the expression of DNA helicase genes and the score of genomic scars are presented in a color scale ranging from red for positive correlation to blue for negative correlation.

**Figure 2:** Box plot of HRD score in BRCA1/2 germline mutated and wild-type breast cancer. The scores for HRD and each type of genomic scar were plotted in three groups of breast cancer patients. Breast cancers patients harboring germline pathogenic were named as “Path” group presented in red. Patients harboring nonpathogenic germline BRCA1/2 mutation were named as “NonPath” group represented in green, while those with germline wild-type BRCA1/2 were named as “WT” group represented in blue.

**Figure 3:** The expression of correlated DNA helicase genes in BRCA1/2 germline mutated breast cancer and in BRCA1/2 wild-type breast cancer with high and low HRD score, respectively. The expression of thirteen significantly correlated genes identified in Figure 1 was plotted in three groups of breast cancer patients. Patients with germline BRCA1/2 mutation were included in the “Patho” group, while patients with germline wild-type BRCA1/2 genes were divided into “WT-High” and “WT-Low” groups according to the score of HRD score.

**Figure 4:** Correlation plot between the predicted HRD score using linear model of DNA helicase genes and the actual HRD score. The horizontal axis displays the HRD score of each individual patients calculated with the expression value of five DNA helicase genes using algorithms developed above, while the vertical axis displays the original HRD score calculated through DNA SNP data.

**Figure 5:** Model for the prediction of HRD phenotype in breast cancer. In breast cancer patients with germline pathogenic BRCA1/2 mutations, cancer cells harbor homologous recombination repair deficiency (HRD) due to malfunction of BRCA1 or BRCA2 protein in DNA damage repair. The application of PARP inhibitors in these patients causes defect in single-strand DNA damage repair due to inhibition of PARP-1 protein. The block of both repair pathways promotes the apoptosis of tumor cells, which is called the “synthetic lethal” mechanism of PARP inhibitors, while for breast cancer patient without pathogenic BRCA1/2 mutations, HRD score can be predicted with gene expression of five DNA helicase genes using the linear regression model to further select breast cancer patients with HRD phenotype. When the predicted score is greater than 0.64, the possibility of HRD should be considered and this part of breast cancer could possibly benefit from the treatment of PARP inhibitors.

## Data Availability

Previously reported data were used to support this study and are available at the TCGA database (https://portal.gdc.cancer.gov/). Other data generated or analyzed during this study are available from the corresponding author upon reasonable request.
